# Comparison of Two Innovative Strategies Using Augmented Reality for Communication in Aesthetic Dentistry: A Pilot Study

**DOI:** 10.1155/2019/7019046

**Published:** 2019-04-03

**Authors:** Romane Touati, Raphaël Richert, Catherine Millet, Jean-Christophe Farges, Irena Sailer, Maxime Ducret

**Affiliations:** ^1^Université de Lyon, Université Lyon 1, Faculté d'Odontologie, Lyon, France; ^2^Hospices Civils de Lyon, Service de Consultations et Traitements Dentaires, Lyon, France; ^3^Division of Fixed Prosthodontics and Biomaterials, University Clinics of Dental Medicine, University of Geneva, Geneva, Switzerland; ^4^Laboratoire de Biologie Tissulaire et Ingénierie thérapeutique, UMR 5305 CNRS/Université Lyon 1, UMS3444 BioSciences Gerland-Lyon Sud, Lyon, France

## Abstract

During dental prosthetic rehabilitation, communication and conception are achieved using rigorous methodologies such as smile design protocols. The aim of the present pilot study was to compare two innovative strategies that used augmented reality for communication in dentistry. These strategies enable the user to instantly try a virtual smile proposition by taking a set of pictures from different points of view or by using the iPad as an enhanced mirror. Sixth-year dental students (*n*=18, women = 13, men = 5, mean age = 23.8) were included in this pilot study and were asked to answer a 5-question questionnaire studying the user experience using a visual analog scale (VAS). Answers were converted into a numerical result ranging from 0 to 100 for statistical analysis. Participants were not able to report a difference between the two strategies in terms of handling of the device (*p*=0.45), quality of the reconstruction (*p*=0.73), and fluidity of the software (*p*=0.67). Even if the participants' experience with the enhanced mirror was more often reported as immersive and more likely to be integrated in a daily dental office practice, no significant increase was reported (*p*=0.15 and *p*=0.07). Further investigations are required to evaluate time and cost savings in daily practice. Software accuracy is also a major point to investigate in order to go further in clinical applications.

## 1. Introduction

In dentistry, smile reconstruction is achieved using rigorous and detailed methodologies which are essential for communication between the practitioner, the laboratory, and the patient [1]. Several protocols were previously proposed, such as the “Digital Smile Design®” (DSD), developed by Christian Coachman [2]. Using only a set of photographs and presentation software, this picture-based strategy (PBS) offers a predictive view of the future patient's smile and makes treatment planning and communication with the patient easier. Until now, protocols have been limited by the following factors: they are handmade or only partly computer-assisted, are two-dimensional (2D), and are only partially immersive for patients. To improve the patient's experience and patient-practitioner communication, clinical protocols and technological evolutions were proposed, such as a mock-up, a video analysis, or a 3D facial conception [2, 3]. These tools provided a better immersivity for patients and additional details for practitioners, who were able to objectively evaluate facial movements in response to emotion and speech. However, all these features are complex to integrate for both the clinician and the laboratory, and they require a significant amount of time, energy, and cost [4].

Technological evolution of hardware and software aims to reduce the time and errors during information sharing between patients, practitioners, and laboratories. The aim of the technology presented in this pilot study is to improve the communication with the patient using facial recognition (FR) and augmented reality (AR). FR is a technology capable of automatically identifying a person from a digital image, using reference lines of the face and mathematical algorithms [5]. AR is a type of technology in which an environment is enhanced through the process of superimposing computer-generated virtual content over a real structure [6, 7]. Even if AR tools are mainly used for video games and animations, the medical field is working to integrate these technologies for diagnosis, surgery, education, and communication with patients [8]. In dentistry, AR was firstly used for educational purposes as a tool to objectively evaluate students and give them direct feedback [8]. However, there is no study that evaluates AR as a tool to improve communication in aesthetic dentistry.

The present pilot study tested the user experiences using two innovative software of augmented reality for communication in aesthetic dentistry; one using a set of pictures and described as an automatized picture-based strategy (APBS), and the other using the front camera system of the touchpad called enhanced mirror strategy (EMS).

## 2. Materials and Methods

In this study, a recent application released for iOS 11 was evaluated, allowing for AR experiences to be created using a recent iPad or iPhone [9–11]. This application (IvoSmile®/Kapanu, Ivoclar-Vivadent) uses the captor camera integrated in a tablet to recognize the patient's face. After having determined virtual facial and oral landmarks [4, 12, 13], a second software proposes an artificial layer of smile propositions that is superimposed on the patient's smile (Figure 1).

Two strategies are possible: the first one (APBS) consists in taking a set of photographs in an automatized version of PBS. The user can instantly change the point of view by scrolling through the different photographs. In the second strategy (EMS), the patient can directly try and modify the proposition by looking at the iPad screen in motion, as an enhanced mirror (Figure 2).

Users can interact and change the shape, size, and color of the teeth using a large range of tools. The software gives the possibility to the user to modify the center of the arch according to the facial midlines (Figure 3(a)) and choose tooth form and proportion within different catalogues of the teeth (Figure 3(b)). The user can also modify the incisal edge position by raising or lowering length and width of the teeth (Figure 3(c)) or by changing the occlusal plane (Figure 3(d)) or the dental arch inclination and width (Figure 3(e)). Finally, the software allows the user to modify the shade and luminosity of the teeth (Figures 3(g)–3(i)).

In the present study, one operator (RT) presented the device to the sixth-year volunteer dental students (18 subjects, women *n*=13, men *n*=5; mean age: 23.8 years). After study subjects provided informed consent, they received some explanation and were requested to freely use the device and the different tools on their own smile (Figure 4).

After ten minutes of use, participants were asked to compare the two strategies (APBS and EMS). The experience of participants while using the application was rated using an anonymous questionnaire and a visual analog scale (VAS). The questionnaire included 5 questions and was adapted from a previous study [3] (Table 1). All supplementary declarative comments of participants were also collected and reported in the present report. VAS answers were converted into a numerical result ranging from 0 to 100 for statistical analysis. A statistical software (IBM SPSS Statistics v24) was used for analyzing data normality. Data were not normally distributed, and a Wilcoxon test was applied to evaluate the difference between the 2 camera systems (*α* = .05).

## 3. Results

18 participants (13 women and 5 men; mean age: 23.8 years) were included in the study. Results of the questionnaire were reported in Table 2. In the present pilot study, participants' preference for one strategy over the other was not significant. Authors were not able to prove a difference between strategies in terms of handling of the device (*p*=0.45), quality of the reconstruction (*p*=0.73), and fluidity of the software (*p*=0.67). According to the participants' experience, EMS was more often reported as immersive, but this study failed to report a significant advantage over the APBS (*p*=0.15). Similarly, participants reported a preference regarding EMS, but the difference was not significant (*p*=0.07). Participants reported that both AR strategies were complementary as they are not used for the same purpose. APBS was described by the participants as a pedagogic tool useful to explain the different smile possibilities to the patient, whereas EMS was used as the virtual try-in phase of the proposed smile project.

## 4. Discussion

The results of the study did not manage to report a significant difference between the two strategies in terms of handling of the device, quality of the reconstruction, fluidity of the software, and immersivity and interest for integration in a daily dental office practice. However, many questions still need to be discussed about this application.

The handling of this innovative software requires a learning curve, and many users reported that the overabundant offer of choices could make the decision process more difficult. Some suggested that the software could be simplified by creating, for example, a step-by-step version of the application, where the user is driven by the software through the different features in a logical and chronological way. Inversely, restricted freedom was reported for the determination of vertical facial and dental midlines, whereas these midlines play a significant role in the smile analysis and differences up to 2-3 mm between facial and dental midlines could be visually noticed [14]. The catalogue of teeth options was also limited, and a deep learning approach could be a valuable way of enhancing the catalogue of the teeth by collecting data from patients' and practitioners' projects.

It has been shown before that mobile devices could serve as an excellent way to communicate in dentistry [3]. Participants reported also a good immersivity for both strategies. These results are close to those of Kim et al., which noted that AR technology was associated with excellent user experiences in education [14]. However, the present work failed to report that immersivity was significantly enhanced using EMS. These results could be explained by the fact that some participants reported a poorer picture quality using EMS, due to the video captor that leads to occasional mismatch or image pixelation. Even if a majority of participants reported their interest in using a similar tool in their daily practice for conception and communication with patients, further investigations are required to evaluate the cost and time savings brought by the device, compared to other PBS such as DSD [2]. It has to be noted that the present pilot study reported only experiences and analysis of the sixth-year students, and it could be interesting to propose this questionnaire to larger amounts of patients and clinicians in order to evaluate the impact of the device in daily professional practice.

Finally, another limitation reported by authors with present APBS or EMS was the impossibility to match the smile design with the digital cast of the patient. Indeed, in order to perform a realistic computer-assisted design (CAD) of the patient prosthesis, the software needs to be highly precise to prevent alignment mistakes during the matching process with the teeth [15]. Moreover, it was impossible to extract data from the software which prevented the analysis of software accuracy. Similar optical systems designed for AR software show a precision close to 5 mm [7]. This accuracy was considered sufficient for clinical applications in maxillofacial surgery, neurosurgery, or surgical endoscopy [16–18]. However, some limitations were reported for these optical systems, and the addition of infrared captors [19–21], structured light, fiducial landmarks [20], or radiopaque markers attached to the patient's skin [22] has been proposed to help the accuracy for facial and dental recognition [5, 7, 22]. Further investigations are then required to evaluate the accuracy of this innovative device and to determine the precision needed in dentistry.

## 5. Conclusion

Although the size of the sample was limited, observations underline a good experience (handling of the device, quality of image, fluidity, and immersion) for users in both techniques. However, no statistically significant difference was observed between the two strategies. Further investigations are required for evaluating the efficacy of such a device in daily practice in particular regarding the economy of time and cost. The software accuracy is also a major point to investigate before going further in clinical practice.

## Figures and Tables

**Figure 1:** Schematic representation showing the basic principles of this technology. After having captured the patient's face with a picture or live with the touchpad camera (a), the FR software recognized virtual landmarks on the face (b), the lips and the smile of the patient (c). The software proposed a first mask on the patient's teeth (d). The overlay of the new mask enabled the visualization of the smile (e), and the patient was able to see the smile projected on the screen, with a set of pictures for APBS or in motion as a mirror in EMS (f).

**Figure 2:** Illustration of the use of the software. (a) Using an iPad camera, the FR software is able to recognize nonfiducial markers (lips, smile, gum, and teeth) (b) and to propose a first mask overlaid on the initial face capture (c). A first smile design proposition is instantly obtained (d).

**Figure 3:** Illustration of some of the different features offered by the software and their impact on the smile rendering. (a) Software determination of the ideal dental midline according to the horizontal and vertical facial midlines, the interpapillary line, and the incisal edge position. (b) Proposition of form from the software catalogue. (c) Determination of the length and width of the teeth. (d)–(f) Determination of the occlusal plan height, inclination, width, and depth of the arch. (g)–(i) The final proposition can be chosen according to luminosity, shade, and color of the teeth.

**Figure 4:** Use of the device. (a) Participant can use the technology by maintaining the tablet at a required minimal distance as a mirror. (b) User can see himself on the screen and interact with the software.

**Table 1:** Questionnaire for participants' perceptions after using APBS and EMS.

Questions for participants	Anchor terms
(1) How do you judge the handling of the device?	(0 = very difficult; 100 = very easy)
(2) How do you judge the quality of the smile reconstruction picture?	(0 = very low; 100 = very high)
(3) How do you judge the fluidity of the software?	(0 = very complicated; 100 = very easy)
(4) Do you find the experience immersive?	(0 = very low; 100 = very high)
(5) Would you be interested in using a similar device in your daily practice?	(0 = no, never; 100 = yes, with pleasure)

**Table 2:** Participants' perceptions of APBS and EMS.

Question	Automatized picture-based strategy			Enhanced mirror strategy			*P*
	Mean ± SD	95% CI	Range	Mean ± SD	95% CI	Range	
1	84 ± 2	80–88	73–100	82 ± 3	76–88	50–100	0.45
2	82 ± 2	77–86	65–100	80 ± 3	73–86	50–100	0.73
3	86 ± 2	81–90	64–100	85 ± 4	77–91	50–100	0.67
4	82 ± 3	75–88	60–100	89 ± 3	84–94	65–100	0.15
5	83 ± 3	76–89	50–100	88 ± 3	80–94	55–100	0.07

## Data Availability

The data used to support the findings of this study are available from the corresponding author upon request.
